The article "Design of Children's Motor Skills Training Management System Based on Human Movement Recognition Algorithm of Depth Information" was retracted in 2023. Reasons: signs of a paper mill; compromised peer review; unreliable results or conclusions.

# Design of Children's Motor Skills Training Management System Based on Human Movement Recognition Algorithm of Depth Information

**DOI:** 10.1155/2022/9618753

**Published:** 2022-03-14

**Authors:** ZhengYi Cheng, Jihui Li

**Affiliations:** ^1^Beijing Sport University, Beijing 100084, China; ^2^Shenyang Sport University, Shenyang 110102, China

## Abstract

With the deepening of the concept of all-round development, the training of children's motor skills is becoming more and more popular. Children's motor skills training management system is based on the product of children's motor skills training combined with modern technology. This article aims to design a management system for children's motor skills training based on human motion recognition methods. This article proposes a human motion recognition algorithm based on depth information. The traditional human motion recognition algorithm is more biased towards children's motor skills. For the design of the system, this article also pays great attention to children's experience. After analyzing the performance of the system in this study, it is found that the system is not ideal for multitarget human motion recognition. Therefore, this article optimizes the recognition. After the optimization, the recognition rate of the head, upper body, and lower body of the multiobjective human motion recognition is more than 80%.

## 1. Introduction

Human body movement is to express a certain will of a person, which includes the movement process or static posture of various parts of the human body, such as hands, feet, head, and body. It is one of the ways that humans interact with the environment. As humans, we have an excellent ability to understand human movement through visual information, and machines currently do not have such performance. Therefore, how to make the machine automatically recognize, understand, and even predict the motion behavior of the human body has become a new focus of attention in the field of computer vision.

The society of training institutions has grown and the competition has become increasingly fierce. Excellent training institutions not only have outstanding internal qualities but also need a sound management mechanism. However, the data management of many training institutions is still manual operation. Only by finding a way out of information management in time can the efficiency of training management be improved. Therefore, at this stage, it is very necessary to propose a design study of children's motor skills training management system based on the depth information of the human body movement recognition algorithm.

This article has several innovations in the design of the system: (1) This article focuses on the analysis of the human body motion recognition algorithm based on depth information. This is of great significance to the design of the subsequent children's motor skills training management system. It can not only perform sports analysis for children's motor skills but also can be extended to other aspects in the future. (2) The design of children's motor skills training management system is divided into three modules: motion detection, motion analysis, and visualization interface. The system of this article is more pure, and the purpose is to maximize the service of children's sports training.

## 2. Related Work

Today's visual tracking algorithms are developing vigorously, and there are constantly new algorithms improving the accuracy, stability, and efficiency of target tracking. However, the field of visual tracking still faces many challenges. How to improve the efficiency of the target tracking algorithm in the following challenges is called the biggest challenge of visual tracking. Choi et al. proposed an algorithm that utilizes multiple filters applied to the entire 3-dimensional input image data set. Through a large number of simulation experiments, they found that compared with traditional algorithms, applying some filters to a certain direction of the 3-dimensional data set can improve the measurement accuracy [1]. Aiming at the problem that it is difficult to balance the speed and accuracy of human behavior recognition, Ju proposed a motion recognition method based on random projection [2]. Li t al. proposed an effective algorithm to solve challenging problems with fast convergence [3]. Xie and Su believed that more and more researchers are beginning to use MEMS sensors to design human motion behavior detection devices. So they studied to determine the motion state of the tested person by tracking the wearer's acceleration changes, and the experimental results show that their method is feasible [4]. Huang and Sun aimed to study 3D human action recognition; their research is very innovative [5]. Ryu et al. conducted research on feature extraction of human lower limbs. Their experimental results show that the average detection accuracy of this method in gait subphase detection, motion pattern recognition, and pattern change detection is better than traditional detection results [6]. Ye et al. proposed a human motion analysis algorithm based on skeleton extraction and a dynamic time warping algorithm based on RGBD camera. The method they proposed can effectively identify single action and double action [7]. Saad analyzed the gait, hoping to conduct biological recognition research through the recognition of the gait. Comprehensive analysis shows that when matched with similar methods in the literature, the proposed algorithm can significantly improve the performance of multiview gait recognition [8]. It can be found that most of the research is to discuss the method and accuracy of recognition, and the application of this aspect to the training of children's sports skills is relatively small.

## 3. Human Motion Recognition Algorithm Based on Depth Information

### 3.1. In-Depth Information

The ways to acquire depth information can be divided into two categories according to the different sensors used: active and passive. The active method uses sensors such as laser, radar, infrared, and ultrasonic to emit energy waves to the measured target and calculates the position of the target by calculating the TOF (Time-Of-Flight) of the energy wave [9, 10]. This type of method has good stability, high accuracy, and fast calculation processing, but the cost of active sensors is high. Some sensors require a special layout environment, are very difficult to use, and are sensitive to the reflection characteristics of the measured object, so this type of method is mainly used in special fields such as military and security. The passive method uses the characteristics of the measured physics itself, such as shape appearance, radiation, and the like, to impose certain physical and geometric constraints to calculate the distance of the object from the observation point. The main methods are angle-based geometric ranging method, target object radiation and atmospheric transmission attenuation method, and image-based ranging method. This kind of method does not need to arrange the signal generator, only needs to use the sensor to collect the characteristic of the measured object itself, it is more convenient to operate. The disadvantage is that the amount of calculation is too large, the stability is low, and the accuracy is lower than that of the active ranging method. This article mainly uses binocular stereo vision to extract the depth information of the scene. This method simulates the principle of the human eye's perception of the scene, imposes constraints on the different positions of the same object in the images captured by the left and right cameras, and then uses the similar triangle formed by the camera and the scene to calculate the distance between the object and the camera. Its advantages are simple system structure, high efficiency, and suitable calculation accuracy. The following will mainly introduce the theoretical basis and specific implementation steps of the release method.

Traditional 2D cameras obtain color information, such as RGB color cameras. The obtained value is the respective pixel value of the three primary colors of red, green and blue, and the size of each pixel value of each channel depends on the light intensity of the lane, such an image contains a lot of texture information and color information, which is greatly affected by illumination factors, and it is difficult for a recognition algorithm based on this to achieve strong robustness. Robustness includes stability robustness and quality robustness. Whether a control system is robust is the key to its actual application. Therefore, the design of modern control systems has taken robustness as one of the most important design indicators. Different from the traditional 2D camera, the depth camera acquires an additional depth image while acquiring the color image, for example, an RGB-D camera adds a depth (Depth) channel to the original RGB three channels of each pixel value, and its value represents the distance of the point in the acquired scene from the camera. The mainstream methods of obtaining depth information are stereo triangulation, time of flight, and structured light [11, 12]. The principles are described below:

#### 3.1.1. Stereo Triangulation Method

The stereo triangulation method is a bionic method inspired by human vision, and its birth can be traced back to the 1960s [13]. It calculates the three-dimensional information of a scene from two or more images collected from different perspectives [14].  Figure 1 shows how the human eye works, using two images collected from two different perspectives to calculate the three-dimensional information of the scene. A point *x* in the scene space is projected to the receiving part *y* of the camera through the focal point *o*, so that the depth information of the point *x* in the scene can be calculated backward when the relative position of the camera is known.

The method of stereo triangulation has low efficiency in extracting depth images from multiple images due to the high complexity of the calculation of the stereo geometry. Moreover, these collected images are sensitive to changes in illumination, which makes the process of matching the triangle relationship more difficult. Due to the main reasons described, the method of using stereo triangulation to extract depth information is difficult to apply to real scenes [15].

#### 3.1.2. Time of Flight Method

Although the three-dimensional triangulation method works well, it does not mean that machines must “see” the world in the same way as humans. To make a method achieve robust results, different sensing technologies can be considered [16, 17]. Different from the stereo triangulation method, camera using time-of-flight method (TOF) emits light pulses directly from a single camera, and the light is reflected back to the camera by the objects in the scene. Then, the machine can calculate the depth information of the scene by combining the time interval between light emission and reception combined with the flight speed of the light.  Figure 2 shows the principle of this method.

Compared with other laser 3D scanning devices, ToF cameras are smaller and cheaper. Most devices on the market today use sinusoidal infrared signals, and the distance information is calculated by a standard CMOS or CCD detector. The mainstream manufacturers of ToF cameras now include PMD and MESA [18]. The advantage of the ToF camera is its high efficiency, and its depth information can cover every pixel (pixel) [19]. The disadvantage is that it is more expensive and has a lower resolution, so fewer researchers or institutions use this type of device.

#### 3.1.3. Structured Light Method

The principle of the structured light method is also based on the triangulation method, but it is different from the stereo triangulation method. As shown in Figure 3, it uses a projector to emit processed light. Most equipment uses raster projection, and then, a camera receives the light reflected by the scene, then compare the received light ripples with the reference ripples calibrated by the system to calculate the depth information of the scene. For example, the values of *a*, *f*, and Z0 in Figure 3 are known, where the reference plane is preset by the system, and the distance between the actual incident point of the reflected light and the default incident point *b* can be converted to obtain the distance Ze between the target and the camera. The principle of the structured light method is simple, the equipment cost is small, and the volume is small. Its limitation is that the measurement result is greatly affected by the system preset value, but this does not affect the method used by the mainstream depth sensor [20, 21].

As shown in Figure 3, the typical camera that adopts the structured light method is the Kinect camera released by Microsoft. Microsoft released Kinect1.0 in 2010 and Kinect2.0 in 2014. Because of its good effects in acquiring depth images and human somatosensory actions and providing open code and program interfaces, many researchers also use it as a depth sensor. In terms of acquiring depth information, Kinect camera is based on the structured light method, which can calculate the depth image of the scene from a single image of reflected light. Its price is low, its size is small, and it is easy to maintain. Nowadays, most of the depth data sets are collected by Kinect. Kinect contains an ordinary RGB camera, an infrared sensor, and a four-microphone array. Combining these devices, Kinect can provide RGB images, depth images and audio signals at the same time.  Figure 4 shows the depth image information generated by Kinect.

### 3.2. Human Motion Recognition Algorithm

In recent years, the technology of image recognition has developed rapidly, and it has a good effect on the recognition of various objects, but it has greater difficulties in the recognition of moving human bodies. The main difficulty lies in (1) the uncontrollable external environment in image acquisition, such as ambient light, background factors, occlusion, and shadows. (2) A good gesture feature description method is the premise of gesture recognition. The uncertainty of attitude makes it difficult to reach a unified index, which increases the difficulty of studying attitude characteristics. (3) The ultimate goal of posture analysis is to understand the information conveyed by a person's posture. This requires not only the recognition of the basic posture of the person but also a comprehensive analysis based on the scene information. At present, a large number of researches are limited to simple types of regular poses, and the analysis of specific poses in specific scenarios needs further research.

Therefore, the main steps of the human body motion recognition algorithm include video image preprocessing, classic background modeling algorithm, and subsequent data processing. Now, we will introduce the human body motion algorithm for these three steps.

#### 3.2.1. Video Image Preprocessing

*(1) Original Image Grayscale*. In order to realize the real-time performance of the algorithm, the original image is converted into a grayscale image before the video image processing, reducing the calculation amount of the algorithm. As the pixels become higher now, the analysis of the original image will be difficult, and the analysis of some colors will increase the amount of calculation, so the image is grayed. In general, the grayscale methods used include component method, maximum value method, average method, and weighted average method.

The component method uses one of the three components of red, green, and blue as the gray value of the pixel, as shown in formula (1):

(1) $$\begin{array}{c} \left\{\begin{array}{c} I=H,\\ I=Lv,\\ I=La. \end{array}\right) \end{array}$$

In formula (1), I represents the pixel brightness of the grayscale image, and H, Lv, and La represent the brightness values of the three components of red, green, and blue. A grayscale image can be selected according to application needs.

The maximum rule takes the maximum value of the three RGB components as the gray value of the pixel, as shown in formula (2). In formula (2), max is the maximum value operation:

(2) $$\begin{array}{c} I=\max\left(H,Lv,La\right). \end{array}$$

The average value rule takes the arithmetic average of the three RGB components as the gray value of the pixel, as shown in formula (3):

(3) $$\begin{array}{c} I=\frac{H+Lv+La}{3}. \end{array}$$

The realization of the maximum value method and the average value method is relatively simple, and the effect is often not good. The grayscale image of the maximum value method is white and lacks contrast. However, the processing performed by the average method will be dark and difficult to extract feature values. Therefore, combining the problems, a weighted average method is proposed. Based on physiological considerations, different weights are assigned to the three components of red, green, and blue. From the perspective of human physiology, the human eye is sensitive to green but insensitive to blue. Therefore, the weighted average method sets the weight of the green component to be larger and the weight of the blue component to be smaller according to the visual model of the human eye, as shown in formula (4). The weights proposed by the OpenCV computer vision open source library are shown in formula (5):

(4) $$\begin{array}{c} I=0.3H+0.5Lv+0.11La, \end{array}$$

(5) $$\begin{array}{c} I=0.2127H+0.7152Lv+0.0722La. \end{array}$$

Generally speaking, the component method and the maximum value method only use one component as the gray value, the form is too single, and the gray image color is too dark or too light. However, the average value method is not based on the visual model of the human eye, and the weight coefficient is unreasonable. From a theoretical and practical point of view, the grayscale effect of the weighted average method is more reasonable and more in line with the needs of practical applications. Therefore, the weighted average method is currently the most commonly used image grayscale method.

*(2) Image Filtering*. Image filtering is one of the indispensable steps in image preprocessing. Its purpose is to maximize the elimination of noise and retain image detail information, laying a good foundation for subsequent processing. The main filtering processing methods are mean filtering, Gaussian filtering, median filtering, and bilateral filtering.

Mean filtering uses the neighborhood averaging method. Assume that the gray values of image pixels (*a*, *b*) before and after filtering are *f*(*x*, *y*, *g*(*a*, *b*)).

The neighborhood template S is an *N* × *N* square window centered on point (*a*, *b*). Finally, the arithmetic average of the gray levels of all pixels in the template neighborhood S is used to replace the gray value of the pixel in the original image, so as to achieve image filtering, which is shown in formula (6):

(6) $$\begin{array}{c} g\left(a,b\right)=\frac{1}{N\times N}\sum_{\left(m,n\right)\leq S}f\left(m,n\right). \end{array}$$

Gaussian filtering, on the basis of neighborhood average, assigns corresponding weights to pixels according to their positions, and takes the weighted average of the gray levels of all pixels in the template neighborhood to replace the gray values of the pixels, so as to achieve image filtering. For example, Figure 5 is a Gaussian template in the 3 × 3 neighborhood, and the pixel weights are sequentially reduced from the center to the periphery, which is more conducive to the preservation of key details of the image.

Median filtering is based on the sorting statistical theory, that is, the gray values of all pixels in a certain pixel neighborhood are arranged in ascending order. It sets its middle value to the gray value of the pixel, so as to remove isolated noise points. Its processing is shown in formula (7):

(7) $$\begin{array}{c} g\left(a,b\right)=\text{Med}\left\{f\left(m,n\right)\right\},\left(m,n\right)\in S. \end{array}$$

Bilateral filtering takes into account both the spatial difference and intensity difference of pixels and takes the weighted average of the gray levels of all pixels in the template neighborhood to replace the gray value of the pixel, as shown in

(8) $$\begin{array}{c} g\left(a,b\right)=\frac{\sum_{k,l}f\left(k,l\right)w\left(m,n,k,l\right)}{\sum_{k,l}w\left(m,n,k,l\right)}, \end{array}$$

(9) $$\begin{array}{c} d\left(m,n,k,l\right)=\exp\left(-\frac{{\left(m-k\right)}^{2}+{\left(n-l\right)}^{2}}{2\sigma_{d}^{2}}\right), \end{array}$$

(10) $$\begin{array}{c} r\left(m,n,k,l\right)=\exp\left(-\frac{{\left\|f\left(m,n\right)-f\left(k,l\right)\right\|}^{2}}{2\sigma_{r}^{2}}\right). \end{array}$$

But its weight coefficient depends on the product of domain kernel formula (9) and value domain kernel formula (10). After the two are multiplied, taking into account the difference between the spatial domain and the value domain at the same time, a data-dependent bilateral filtering weight function is generated as shown in

(11) $$\begin{array}{c} w\left(m,n,k,l\right)=\exp\left(-\frac{{\left(m-k\right)}^{2}+{\left(n-l\right)}^{2}}{2\sigma_{d}^{2}}-\frac{{\left\|f\left(m,n\right)-f\left(k,l\right)\right\|}^{2}}{2\sigma_{r}^{2}}\right). \end{array}$$

#### 3.2.2. Classical Background Modeling Algorithm

The focus of background subtraction is to achieve background modeling. Commonly used modeling algorithms include mean or median filter method, nonparametric method, single Gaussian background modeling method, and mixed Gaussian background modeling method. Among them, the most successful application is mixed Gaussian background modeling. Its main idea is to use K single Gaussian distribution states to represent each pixel and to match these models one by one during detection, which can handle multiple background changes at the same time. Generally, the K value is 3–7.

Assuming that *A*_*t*_ represents the pixel value at time t, formula (12) is the weighted sum of the probability density functions of the N Gaussian models established:

(12) $$\begin{array}{c} P\left(A_{t}\right)=\sum_{i=1}^{N}w_{i,j}\times \eta \left(A_{i},u_{i,j},\sum_{i,j}\right). \end{array}$$

In the formula, represent the weight, mean, and covariance matrix of the *i*-th model at time *t*, where the probability density function is as in

(13) $$\begin{array}{c} \eta \left(A_{i},u_{i,j},\sum_{i,j}\right)=\frac{1}{{\left(2\pi \right)}^{\pi /2}{\left|\sum_{i,j}\right|}^{1/2}}e. \end{array}$$

When a new frame of video image comes, the pixel value *I* (*x*, *y*) of each point in the current frame and the established K Gaussian models of the pixel point are sequentially matched and tested, as shown in formula (14):

(14) $$\begin{array}{c} \left|I_{t}\left(a,b\right)-u_{i,t-1}\right|<D\times \sigma_{i,t-1}, \end{array}$$

where *D* represents the confidence parameter. For the successfully matched model, the parameter update will be completed. The update process is as shown in formulas (15), (16), and (17):

(15) $$\begin{array}{c} w_{i,t}=\left(1-\alpha \right)\times w_{i,t-1}+\alpha , \end{array}$$

(16) $$\begin{array}{c} u_{i,t}=\left(1-\rho \right)\times u_{i,t-1}+\rho \times A_{t}, \end{array}$$

(17) $$\begin{array}{c} \sigma_{i,t}^{2}=\left(1-\rho \right)\times \sigma_{i,t-1}^{2}+\rho \times {\left(A_{t}-u_{i,t}\right)}^{T}\times \left(A_{t}-u_{i,t}\right). \end{array}$$

If the matching is unsuccessful, just update the weights according to formula (18), and the mean and variance remain unchanged.

(18) $$\begin{array}{c} w_{i,t}=\left(1-\alpha \right)\times w_{i,t-1}. \end{array}$$

In the above formula, *α* is the weight learning rate, and *β* is the parameter learning rate.

Compared with the foreground, the background stays in the image for a longer time, and its weight is larger, so the model with larger weight can be regarded as the best description model, as in

(19) $$\begin{array}{c} B=\arg\;\min_{b}\left(\sum_{k=1}^{b}w_{k}>T\right). \end{array}$$

Among them, *T* is the background threshold, usually 0.8. Repeat the steps, if the current frame I (*a*, *b*) and any one of the B models are successfully matched, the pixel is judged as a background point; otherwise, it is judged as a front spot, that is, a moving target. The specific identification process is shown in Figure 6.

## 4. Design of Children's Sports Skills Training Management System

The system is based on the principle of geometric affine 3D image reconstruction. The experimental design of this article chooses to use Kinect sensor as the device to obtain depth information and use ordinary computer to perform image preprocessing, camera calibration, point cloud registration, point cloud stitching, point cloud fusion, and registration visualization with the data information captured by Kinect. Finally, it can see the three-dimensional model of the object to be tested, the overall experimental equipment requirements are low, and the platform is easy to build. The three-dimensional surface reconstruction of the target object is realized through the three-dimensional reconstruction software development platform in the PC, and the visualization of the reconstructed model is realized.

Developers can use the KinectSDK provided by Microsoft to obtain the target's in-depth data. KinectforWindowsSDK can greatly reduce the development threshold of Kinect applications. Developers do not need to pay attention to the cumbersome data exchange process in sensors and middleware, they only need to master the basic SDK and Windows programming to develop related applications. The specific system framework is shown in Figure 7.

### 4.1. Motion Monitoring Module

The exercise monitoring module is the data collection module of the system. In the children's exercise training process, the data during the training process must be recorded.

Video target tracking is a way of using a computer to imitate the human visual perception mechanism, paying attention to an object in the field of view. A machine learning algorithm that searches for the exact position of the target in each frame of the video sequence through an algorithm and uses a visual frame to mark the target. Most target tracking algorithms use a single feature of the color image to describe the appearance of the target. However, the single feature description ability has certain limitations. It is easy to cause the algorithm to be affected under complex environmental changes, and the target location mark is prone to drift and even leads to tracking failure. CT algorithm and fast compression tracking algorithm use randomly selected compression features in the target frame to achieve tracking. However, the Haar-like features extracted from color images are easily affected in complex environments and pose challenges to the accuracy and robustness of target tracking results. Meanshift tracking (meanshift) algorithm uses color histograms to build a target appearance model. The similarity and color characteristics of the target foreground and background are unstable under light changes. When the tracking algorithm uses unreliable features to search and update the algorithm, it is easy to cause drift problems and even lose the target.

### 4.2. Motion Analysis

Constructing the imaging model of the depth camera is to describe the relationship between the optical characteristics and the image of the depth camera through an accurate mathematical model. The measurement modeling of the depth camera is mainly composed of two parts: one part is the same as the ordinary RGB camera, which determines the pixel coordinates through the pinhole model; the other part determines the value of the pixel coordinates through the time-of-flight principle.

As shown in Figure 8, the body joints are divided into 3 parts, the head, the upper body, and the lower body. The video recording of sports training is carried out through the camera, and then the joint information of the video is extracted for simulation analysis to meet the design requirements of the children's sports skill training management system.

## 5. System Performance Analysis

### 5.1. Image Processing Analysis

#### 5.1.1. Analysis of Filtering Effect

Normalized mean square error NMSE and peak signal-to-noise ratio PSNR are generally used to evaluate the effect of image processing.

(20) $$\begin{array}{c} \text{NMSE}=\frac{\sum_{m=0}^{N}\sum_{n=o}^{M}{\left(g\left(m,n\right)-f\left(m,n\right)\right)}^{2}}{\sum_{m=0}^{N}\sum_{n=0}^{M}f{\left(m,n\right)}^{2}}, \end{array}$$

(21) $$\begin{array}{c} \text{PSNR}=\frac{MAX^{2}\times M\times N}{\sum_{m=0}^{N}\sum_{n=0}^{M}{\left(g\left(m,n\right)-f\left(m,n\right)\right)}^{2}}. \end{array}$$

NMSE is shown in formula (20), which represents the denoising ability of the algorithm. PSNR is shown in formula (21), which represents the ability of the algorithm to protect image details. The larger their value, the stronger the algorithm performance. In formula (21), *M* and N are the length and width of the image; MAX represents the maximum gray value of the pixel in the image, usually 255. *f*(*m*, *n*) and *g*(*m*, *n*) are the gray values of the image before and after filtering, respectively.

When processing with a 3 × 3 window template, the filter parameters of different filter methods are shown in Table 1. It can be obtained by comparison: the mean filtering algorithm is simple and easy to implement, and the time consumption is minimal. The median filter is less affected by noise and has the strongest denoising ability. Bilateral filtering has the strongest detail protection capability. Based on the requirements of the real-time performance of the system and the requirements of the algorithm for the completeness of the image edge information, this article chooses the bilateral filtering algorithm.

#### 5.1.2. Analysis of Multitarget Recognition Effect

In actual scenarios, it is generally multiobjective because children's skill training is group based, and one-to-one teaching is less, so systematic multiobject recognition should be studied.

Heterogeneous Earliest Finish Time (HEFT) algorithm is the most well-known DAG scheduling algorithm in the industry due to its good performance and low complexity. The algorithm selects the task with the highest rank value at each step and assigns the selected task to the corresponding processor.  Table 2 shows the priority values of tasks in the DAG.

Finally, these tasks are {n1, n3, n4, n2, n5, n6, n9, n7, n8, n10} according to the scheduling order of the HEFT algorithm. After sorting, it has a good effect on task execution and can save system identification time.

Table 3 is the execution time. For example, the values 13, 19, and 18 in the second row represent the time for task n1 to execute at the maximum frequency on processors u1, u2, and u3, respectively.

It can be seen from Table 3 that the reaction time of the recognition system for different targets is different, and different processors have different recognition efficiency for different targets. Therefore, it is necessary to analyze the recognition efficiency of the system for this situation.

### 5.2. System Identification Efficiency Analysis

First, use the method of extracting skeleton joint point data described in this chapter to extract the skeleton joint point data of the action sequence in MSR-Action3D that uses the depth map sequence as the storage method. We divide the extracted data points into three parts, namely, the head (P1), the upper body (P2), and the lower body (P3). It analyzes the recognition efficiency of the feature extraction of these three parts and finally obtains the experimental results as shown in Table 4.

From the experimental results, we can see that in the analysis of the skeleton joint point data of the data set, the system has the highest recognition efficiency for the head, with an average value of 88.16%. The effect for the upper body is not much different from that of the head, at 88.05%, but the recognition effect for the lower body is slightly lower, only reaching 72.98%. The preliminary judgment is because there are more joints in the lower body, which puts a lot of pressure on the recognition of the system, resulting in a slightly lower accuracy.

Then, the recognition efficiency of different numbers of people was tested, and five sets of video data with children's skill training as 1, 5, 10, 15, and 20 were selected for recognition. The results are shown in Figure 9.

As shown in Figure 9, in the multitarget recognition, the recognition efficiency of the head will not decrease with the increase of the number of recognition, and it has been around 88%. The recognition efficiency of the upper body and the lower body will decrease with the increase of the number of people, especially the lower body, with the increase of the number of people, it will decrease at a rate of about 2%, and it will decrease to 60% for about 20 people. So for this phenomenon, we need to optimize it. It is mainly optimized on the joint points of the three parts, combining the joints of the head and shoulders and combining the joint points of the lower body with the upper body. The optimization result is shown in Figure 10.

As shown in Figure 10, the accuracy of multitarget recognition has been greatly improved after optimization. Especially in the optimization of the lower body, the recognition efficiency has increased by 23%, an increase of about 50%. Therefore, the optimized body joint partition is more suitable for the feature extraction and validity recognition of the system.

## 6. Conclusions

Today, everything is developing in the direction of intelligence. The children's motor skills training management system studied in this article is an intelligent platform for children's training. This article first briefly introduces the background of the article and then makes relevant explanations about relevant research at home and abroad. It is believed that relevant work is more about describing the efficiency and accuracy of human movement recognition, but there is no relevant research for children. After that, the article gives a detailed introduction to the extraction of depth information and the human motion recognition algorithm to pave the way for the design of the article system. Later, the article system is designed, which is mainly divided into motion monitoring, motion analysis, and visualization interface. The system is very simple and meets the needs of children. Finally, this article analyzes the performance of the design system. The experimental results believe that the recognition efficiency of the system can reach more than 80%. But there are also shortcomings in this article. In subsequent articles, the design of the system will be strengthened and certain functions will be added.

## Figures and Tables

**Figure 1:** An example of the principle of stereo triangulation.

**Figure 2:** Example of the principle of the time-of-flight method.

**Figure 3:** The principle of structured light ranging and Kinect 2.0 released by Microsoft.

**Figure 4:** Original image and generated IR and image depth map.

**Figure 5:** Gaussian template.

**Figure 6:** Flow chart of human motion image extraction algorithm.

**Figure 7:** Children's motor skills training management system.

**Figure 8:** Feature descriptor example.

**Figure 9:** Accuracy of multitarget recognition.

**Figure 10:** Comparison of recognition rates before and after optimization.

**Table 1:** Quality comparison of various filtering methods.

Filtering method	Time-consuming (ms)	NMSE/10^−3	PMSR
Mean filter	1.29391	3.7342	29.9111
Gaussian filtering	2.82287	3.21919	30.5556
Median filter	19.0608	4.36952	29.2288
Bilateral filtering	5.05562	0.0173025	53.252

**Table 2:** Priorities corresponding to each task.

Task	Rank
n1	108
n2	70
n3	80
n4	80
n5	69
n6	63.3
n7	42.7
n8	35.7
n9	44.3
n10	14.7

**Table 3:** The parameters of the processor for each subtask in the application.

Task	u1	u2	u3
n1	14	16	9
n2	13	19	18
n3	11	13	19
n4	13	8	17
n5	12	13	10
n6	13	16	9
n7	7	15	11
n8	5	11	14
n9	18	12	20
n10	21	7	16

**Table 4:** Results of the system's single joint recognition experiment.

	P1 (%)	P2 (%)	P3 (%)
Test 1	88.42	86.62	73.14
Test 2	86.68	85.93	81.29
Test 3	89.39	91.62	64.52
Mean	88.16	88.05	72.98

## Data Availability

The data sets used and/or analyzed during the current study are available from the corresponding author on reasonable request.

## References

[1] Choi I. H., Kim J. S., Joo H. (2017). Study on multi-plane extended depth of focus algorithm for three dimensional information extraction. *Journal of Institute of Control Robotics & Systems*.

[2] Ju Y. (2021). Study of human motion recognition algorithm based on multichannel 3D convolutional neural network. *Complexity*.

[3] Li Z., Nie F., Chang X., Yang Y. (2017). Beyond trace ratio: weighted harmonic mean of trace ratios for multiclass discriminant analysis. *IEEE Transactions on Knowledge and Data Engineering*.

[4] Xie Y., Su H. (2018). Application and research of mems sensor in gait recognition algorithm. *Paper Asia*.

[5] Huang R., Sun M. (2021). Network algorithm real-time depth image 3D human recognition for augmented reality. *Journal of Real-Time Image Processing*.

[6] Ryu J., Lee B. H., Kim D. H. (2017). sEMG signal-based lower-limb human motion detection using top and slope feature extraction algorithm. *IEEE Signal Processing Letters*.

[7] Ye Q., Qu C., Zhang Y. (2018). Human motion analysis based on extraction of skeleton and dynamic time warping algorithm using RGBD camera. *International Journal of Applied Pattern Recognition*.

[8] Saad M. (2017). Design of adaptive biometric gait recognition algorithm with free walking directions. *IET Biometrics*.

[9] Zhang X. (2021). Application of human motion recognition utilizing deep learning and smart wearable device in sports. *International Journal of System Assurance Engineering and Management*.

[10] Qin T., Yang Y., Wen B. (2021). Research on human gait prediction and recognition algorithm of lower limb-assisted exoskeleton robot. *Intelligent Service Robotics*.

[11] Saleh A. M., Hamoud T. (2021). Analysis and best parameters selection for person recognition based on gait model using CNN algorithm and image augmentation. *Journal of Big Data*.

[12] Zhang D. (2021). Intelligent recognition of dance training movements based on machine learning and embedded system. *Journal of Intelligent and Fuzzy Systems*.

[13] Kumar P., Mukherjee S., Saini R., Kaushik P., Roy P. P., Dogra D. P. (2019). Multimodal gait recognition with inertial sensor data and video using evolutionary algorithm. *IEEE Transactions on Fuzzy Systems*.

[14] Wang Y., Wang W., Tian S., Li P. (2018). Human motion recognition based on electrostatic signals. *Jiqiren/Robot*.

[15] Zhu M., Huang Q. (2017). Research on 3D human motion analysis and action recognition method. *Revista de la Facultad de Ingenieria*.

[16] Sepahvand M., Abdali-Mohammadi F., Mardukhi F. (2017). Evolutionary metric-learning-based recognition algorithm for online isolated Persian/Arabic characters, reconstructed using inertial pen signals. *IEEE Transactions on Cybernetics*.

[17] Kumar N., Sukavanam N. (2018). Motion trajectory for human action recognition using fourier temporal features of skeleton joints. *Journal of Image and Graphics*.

[18] Zhu G. Z., Wang Y. X. (2017). Research on human body motion attitude capture and recognition based on multi-sensors. *Revista de la Facultad de Ingenieria*.

[19] Zha S., Li T., Cheng L. (2021). Exoskeleton follow-up control based on parameter optimization of predictive algorithm. *Applied Bionics and Biomechanics*.

[20] Fang H., Tang P., Si H. (2020). Feature selections using minimal redundancy maximal relevance algorithm for human activity recognition in smart home environments. *Journal of Healthcare Engineering*.

[21] Liao S., Li G., Li J. (2020). Multi-object intergroup gesture recognition combined with fusion feature and KNN algorithm. *Journal of Intelligent and Fuzzy Systems*.

